This article has been retracted.

# Progesterone and calcitriol reduce invasive potential of endometrial cancer cells by targeting ARF6, NEDD9 and MT1-MMP

**DOI:** 10.18632/oncotarget.22745

**Published:** 2017-11-28

**Authors:** Sana Waheed, Batsukh Dorjbal, Chad A. Hamilton, G. Larry Maxwell, Gustavo C. Rodriguez, Viqar Syed

**Affiliations:** ^1^ Uniformed Services University, Department of Obstetrics and Gynecology, Bethesda, MD 20814, USA; ^2^ Women’s Health Integrated Research Center at Inova Health System, Department of Defense Gynecologic Cancer Center of Excellence, Annandale, VA 22003, USA; ^3^ John P. Murtha Cancer Center at Water Reed National Military Medical Center, Bethesda, MD 20889, USA; ^4^ Inova Fairfax Hospital, Department of Obstetrics and Gynecology, Falls Church, VA 22042, USA; ^5^ Division of Gynecologic Oncology, North Shore University Health-System, University of Chicago, Evanston, IL 60201, USA; ^6^ Uniformed Services University, Department of Molecular and Cell Biology, Bethesda, MD 20814, USA

**Keywords:** migration, invasion, matrix metalloproteinases, invadopodia, membrane trafficking

## Abstract

Previously, we have demonstrated that progesterone and calcitriol synergistically inhibit growth of endometrial and ovarian cancer by enhancing apoptosis and causing cell cycle arrest. Metastasis is the main reason of mortality in cancer patients. Activation of ADP-Ribosylation Factor 6 (ARF6), Neural Precursor cell expressed Developmentally Downregulated 9 (NEDD9), and Membrane-Type-1 Matrix Metalloproteinase (MT1-MMP) have been implicated in promoting tumor growth and metastasis. We examined the effects of progesterone, calcitriol and progesterone-calcitriol combination on metastasis promoting proteins in endometrial cancer. Expression of ARF6, NEDD9, and MT1-MMP was enhanced in advanced-stage endometrial tumors and in cancer cell lines compared to normal tissues and immortalized EM-E6/E7-TERT endometrial epithelial cells. Knockdown of these proteins significantly inhibited the invasiveness of the cancer cells. The expression levels of all three proteins was reduced with progesterone and progesterone-calcitriol combination treatment, whereas calcitriol alone showed no effect on their expression but moderately decreased MT1-MMP activity. Fluorescence microscopy showed membrane expression of MT1-MMP in vehicle and calcitriol-treated endometrial cancer cells. However, progesterone and calcitriol-progesterone combination treatment revealed MT1-MMP in the cytoplasm. Furthermore, progesterone and calcitriol reduced the activity of MT1-MMP, MMP-9, and MMP-2. In addition, invadopodia regulatory proteins were attenuated in both progesterone and progesterone-calcitriol combination treated cells as well as in MT1-MMP knockdown cells. Thus, targeting the aberrant MT1-MMP signaling with progesterone-calcitriol may be a novel approach to impede MT1-MMP mediated cancer dissemination and may have therapeutic benefits for endometrial cancer patients.

## INTRODUCTION

Tumor cells have the tendency to move from a primary site to distant organs, eventually causing cancer associated death. The metastatic cascade has three steps: invasion, intravasation, and extravasation. The loss of cell-cell adhesion allows tumor cells to detach from the primary tumor mass. Metastatic cells have high levels of proteolytic enzymes, called matrix metalloproteinase (MMPs), which are capable of degrading extracellular matrix (ECM) components, resulting in ruptured tissue barriers and invasion of cells to surrounding stroma. To disseminate to other organs, cancer cells invade the vasculature of neighboring normal tissues or the neovasculature of the tumor, then move to distant sites and form new metastatic colonies [1, 2].

The ADP-ribosylation factors (ARFs) belong to a family of Ras related GTP-binding proteins. They are implicated in tumor angiogenesis, growth, invasion, and metastasis. Six types of mammalian ARFs work as switches between GDP-bound inactive and GTP-bound active states. ARFs 1-5 are localized on Golgi complex and endoplasmic reticulum and control membrane trafficking between these two intracellular organelles. ARF6, which is present on the plasma membrane and endosomes, facilitates membrane ruffle formation, endocytosis and exocytosis of different receptors, modulation of cell adhesion molecules and plays a crucial role in cancer growth, invasion and metastasis [3–7].

Similar to ARF6, the neural precursor cell expressed developmentally down regulated 9 (NEDD9) is also implicated in tumor invasion and metastasis. Several studies correlate elevated levels of NEDD9 with poor tumor prognosis [8–10]. The function of NEDD9 in tumorigenesis is supported by enhanced SNAIL, SLUG, vimentin and decreased E-cadherin expression [11–13]. Furthermore, NEDD9 silencing is associated with attenuated cancer growth and enhanced apoptosis [13, 14].

The MMPs are highly expressed in metastatic cancers and correlate with poor survival. Based on peptide domain structure, amino acid sequence and substrate specificity, MMPs are categorized into twenty-three types. Their function is to break down multiple substrates in the extracellular matrix and they are implicated in tumor invasion, metastasis, and angiogenesis [2, 15]. In addition to secreted MMPs, there are six types of membrane-type (MT) MMPs. These matrix metalloproteinases have membrane-anchoring domains that place them at the cell surface [15]. MT1-MMP, a transmembrane metalloproteinase, is produced in cells as a latent∼72-kDa zymogen. It is activated by a Golgi-associated subtilisin-like serine proteinase furin, into a ∼60-kDa catalytically active protease [16, 17]. MT1-MMP is upregulated in a number of cancers, degrades fibrillar collagens types I, II, and III and plays a pivotal role in tumor growth, invasion, and angiogenesis [18–21]. MT1-MMP is internalized from the cell surface in clathrin- and caveolae-dependent manners in early and late endosomes, where a part of the enzyme is either autodegraded or recycled back to the cell surface to develop new invadopodia [22–25] facilitating the migration of cells.

NEDD9 and ARF6 are shown to be involved in trafficking of MT1-MMP, which via modulation of invadopodia, eventually affects tumor metastasis [26]. Invadopodia are membrane projections of cancer cells that degrade the extracellular matrix and have a key role in cancer invasion and metastasis. Several studies have demonstrated that endocytic and exocytic trafficking is essential for the transport of MT1-MMP to invadopodia. The accumulation of MT1-MMP on the surface of cell results in formation of invadopodia and contributes to their proteolytic activity. Invadopodia have several proteins that are grouped based on their cellular functions: motility associated proteins (N-WASP, cortactin, Arp2/3, Nck, Cdc42, cofilin, dynamin and capping proteins), adhesion proteins (integrins), signaling proteins (tyrosine kinases and Ras-related GTPases) and membrane-associated proteases (MT1-MMP, MMP-2, MMP and the urokinase-type plasminogen activator (uPA)/uPA receptor proteolytic system).

A recent study by Loskutov et al, [26] demonstrated that NEDD9 decreased levels of ARF6, perturbed trafficking of MT1-MMP, and subsequently decreased tumor invasion and metastasis. While high expression levels of ARF6, NEDD9 and MT1-MMP have been suggested to support tumor metastasis, no evidence to date has shown whether and how they influence endometrial cancer metastasis.

In our previous studies, we have shown that combining progesterone with calcitriol have synergistic inhibitory effects on growth of endometrial and ovarian cancer cells [27–30]. The aim of the present study is to evaluate whether the combination of progesterone with calcitriol exerted antitumor effects on invasion and metastasis of human endometrial cancer cells. In this study, we demonstrated overexpression of all three proteins in endometrial cancer and attenuation of their expression by progesterone/calcitriol which resulted in a marked reduction in the expression of invadopodia formation proteins, and thus inhibition of tumor metastasis.

## RESULTS

### ARF6, NEDD9 and MT1-MMP expression is increased with tumor progression

The TMAs (US Biomax Inc.) comprised of 12 normal and 59 malignant tissues were used to analyze the expression of ARF6, NEDD9 and MT1-MMP by immunohistochemistry. On TMAs, there were 22, 20 and 17 tissues from grade I, grade II, and grade III cancers respectively. The levels of ARF6, NEDD9 and MT1-MMP were low to undetectable in normal endometrial tissues. However, high levels of ARF6, NEDD9 and MT1-MMP were detected in grade II and grade III tumors (Figure 1 and Table 1). The data correlated enhanced expression of ARF6, NEDD9, and MT1-MMP with endometrial carcinogenesis. We also compared the expression of ARF6, NEDD9 and MT1-MMP, in three endometrial cancer cell lines and an immortalized endometrial epithelial cell line. Compared to EM-E6/E7-TERT cells, endometrial cancer cell lines expressed the three proteins at higher levels (Figure 2). The expression pattern of the three proteins in cell lines corroborated with the expression pattern in TMAs.

**Figure 1:** Expression of ARF6, NEDD9 and MT1-MMP is associated with endometrial tumor progression ARF6, NEDD9 and MT1-MMP protein levels were analyzed in tissue microarrays using immunohistochemistry. Levels of all the three proteins were higher in Grade III tumors than in normal endometrial tissues. Negative controls for ARF6, NEDD9 and MT1-MMP are shown in Grade III tumor tissue. Original magnification, 400x.

**Table 1:** Correlation between clinicopathologic feature of patients and intensity of ARF6, NEDD9 and MT1-MMP

	Clinical Parameters					Cores (%)		
Tissues	Grade	Age (y)	Tumor	Cores	Staining	ARF6	NEDD9	MT1-MMP
Normal	NA	37–72	NA	23	Low (1–2)	94.34 ± 0.11	95.45 ± 0.21	97.40 ± 0.21
					High (3–4)	5.66 ± 0.18	4.55 ± 0.11	3.59 ± 0.27
Malignant	Gr .I	36–57	T1. T2	60	Low (1–2)	25.56 ± 0.21	17.45 ± 0.32	20.23 ± 0.21
					High (3–4)	**74.44 ± 0.19**	**82.55 ± 0.19**	**79.77 ± 0.32**
	Gr .II	29–84	T1. T2	120	Low (1–2)	14.98 ± 0.22	10.56 ± 0.24	15.07 ± 0.27
					High (3–4)	**85.02 ± 0.15**	**89.03 ± 0.11**	**84.93 ± 0.19**
	Gr. III	45–80	T1. T2 T3. T4	34	Low (1–2)	10.78 ± 0.12	9.65 ± 0.13	11.30 ± 0.45
					High (3–4)	**89.22 ± 0.22**	**90.44 ± 0.18**	**88.68 ± 0.36**

NOTE: Grade I, indicates well differentiated; Grade II, moderately differentiated; Grade III, poorly differentiated; T1, indicates tumor invades submucosa; T2, tumor invades muscularis propria; T3, tumor invades through muscularis propria into subserosa or into nonperitonealized pericolic or perirectal tissues; T4, tumor directly invades other organs or sturtures and/or perforate. Staining intensity: 0, no staining; 1, weak; 2, moderate; 3, strong. The percentage of cells expressing elevated levels of ARF6, NEDD9 and MT-MMP was high in endometrial tumors compared to normal endometrium. Statistically significant (*p* < 0.05) values are given in bold.

**Figure 2:** Expression of ARF6, NEDD9 and MT1-MMP in immortalized endometrial epithelial EM-E6/E7/TERT cells and endometrial cancer lines Immortalized EM-E6/E7/TERT and endometrial cancer cell lines (HEC-1B, Ishikawa, and RL-95) were evaluated by Western blot for basal expression of ARF6, NEDD9 and MT1-MMP. β-actin was used as a loading control. Representative Western blot analyses of 3 independent experiments with similar results are shown. The values above the bands represent relative density of the bands normalized to β-actin.

### Expression of ARF6, NEDD9 and MT1-MMP is associated with cancer cell invasiveness

The invasive potential of HEC-1B and Ishikawa cells was examined in ARF6, NEDD9 and MT1-MMP knockdown cancer cells and their counterpart scrambled siRNA transfected cells. The expression of ARF6, NEDD9 and MT1-MMP was markedly reduced in siRNA-ARF6, siRNA-NEDD9 and siRNA MT1-MMP transfected cells respectively (Figure 3A). We also examined the effect on protein knockdown on cell invasiveness. ARF6, NEDD9 and MT1-MMP knockdown cells showed significantly reduced invasive potential compared with ARF6, NEDD9 and MT1-MMP expressing cells (Figure 3B). These results suggest that all the three proteins play an important role in cell migration and invasion.

**Figure 3:** Effect of ARF6, NEDD9 and MT1-MMP silencing on protein expression and invasiveness of malignant cells Cells were transfected with ARF6, NEDD9 and MT1-MMP siRNAs (25 nmol/L) or scrambled siRNA (25 mmol/L) using Dharmafect. (**A**) Expression of ARF6, NEDD9 and MT1-MMP was analyzed by Western blot analysis. The values above the bands represent relative density of the bands normalized to β-actin. (**B**) Cells invasive potential was evaluated by using Matrigel Invasion Chambers. Data shown are mean ± SEM of values from 3 independent experiments. Statistically significant changes in the ARF6, NEDD9 and MT1-MMP knockdown groups compared to their respective control groups are shown by asterisk (*P* < 0.05).

### Progesterone and calcitriol attenuates ARF6, NEDD9 and MT1-MMP expression in endometrial cancer cells

The effect of progesterone and calcitriol on ARF6, NEDD9 and MT1-MMP expression in HEC-1B and Ishikawa cells was examined. Progesterone in combination with calcitriol significantly reduced expression of all three proteins in both cell lines. Inhibition was more distinct in cells treated with combination treatment than with progesterone alone. Calcitriol alone had no marked effect on ARF6, NEDD9 and MT1-MMP expression (Figure 4A). To confirm that progesterone inhibits expression of these three proteins, cells were cultured with progesterone, calcitriol or the combination in the presence or absence of progesterone receptor antagonist (mifepristone RU 486). Progesterone failed to reduce ARF6, NEDD9 and MT1-MMP expression in both cell lines exposed to progesterone and its antagonist (Figure 4B). These results suggest that progesterone can successfully attenuate expression of proteins participating in cancer cell invasion.

**Figure 4:** Expression of ARF6, NEDD9 and MT1-MMP in endometrial cancer lines (**A**) HEC-1B and Ishikawa cells were treated with progesterone (PROG, 20 µmol/L), calcitriol (CAL, 100 nmol/L) or combination for 72 h were evaluated by Western blot analysis for expression of ARF6, NEDD9 and MT1-MMP. (**B**) To confirm the specificity of PROG, cells were treated as stated above in the presence of progesterone antagonist (0.1 mM, RU 486) for 72 h and evaluated for the expression of ARF6, NEDD9 and MT1-MMP by Western blotting. Representative Western blot analyses of 3 independent experiments with similar results are shown. The values above the bands represent relative density of the bands normalized to β-actin.

### Progesterone affects localization of MT1-MMP in cancer cells

MT1-MMP has a critical role in tumor progression and metastasis. Upon accumulation of MT1-MMP on the surface of cells, it instigates formation of invadopodia that are implicated in tumor cell invasion and dissemination. Therefore, the effect of progesterone, calcitriol and their combination on the subcellular localization of MT1-MMP in HEC-1B and Ishikawa cells was examined. The results for HEC-1B cells are shown (Figure 5A). In vehicle treated cells, MT1-MMP was localized on the cell membrane. Progesterone treatment of cells reduced abundance of cell surface localized MT1-MMP and translocated it from the membrane to the cytoplasm. Calcitriol exhibited no effect on MT1-MMP translocation. Progesterone and calcitriol combination was able to translocate MT1-MMP to the cytoplasm. Quantitative analysis of the fluorescence showed high expression of MT1-MMP in vehicle and calcitriol treated cells compared to progesterone treated cells. Treatment of cells with progesterone and calcitriol combination further decreased MT1-MMP expression compared to progesterone alone treated cells (Figure 5B). Together, these data suggest that progesterone-calcitriol combination by reducing MT1-MMP expression and translocating it from cell membrane to the cytoplasm attenuates invasive potential of cells.

**Figure 5:** Localization of MT1-MMP in HEC-1B cells (**A**) Cells were treated with progesterone (PROG, 20 µmol/L), calcitriol (CAL, 100 nmol/L) or combination for 24 hours. The cell images were aligned into four vertical panels: the first vertical panel shows nuclear staining with DAPI, the second shows MT1-MMP signal, the third shows F-actin staining and the fourth is the overlay of DAPI, MT1-MMP and F-actin. (**B**). The intracellular MT1-MMP pixel values measured in confocal z-stacks using Image J. Thirty cells were measured for each treatment group. The expression of MT1-MMP was significantly less in progesterone and calcitriol-progesterone groups compared to vehicle treated cells (^*^P < 0.05).

### Progesterone and calcitriol reduced activity of MT1-MMP in endometrial cancer cells

After establishing that progesterone and its combination with calcitriol reduced the expression of MT1-MMP, we were interested in determining whether the two agents affect its activity. About 15–20% inhibition of MT1-MMP activity was demonstrated in calcitriol alone treated cells compared to vehicle treated cells. Progesterone treatment attenuated 53–67% of MT1-MMP activity in HEC-1B and Ishikawa cells respectively compared to vehicle treated cells. Progesterone and calcitriol combination treatment suppressed MT1-MMP activity between 63 and 76% in HEC-1B and Ishikawa cells respectively compared to vehicle treated cells. Progesterone- calcitriol combination reduced MT1-MMP activity by 10% in HEC-1B and 9% in Ishikawa cells compared to progesterone alone treated cells (Figure 6A). Since MT1-MMP is an activator of MMP-9 and MMP-2, we also analyzed their activities in progesterone-calcitriol treated cells. Exposure of cells to calcitriol decreased MMP-9 activity by 19% in HEC-1B and 23% in Ishikawa cells compared to vehicle treated cells. HEC-1B and Ishikawa cells showed 57% and 62% decrease in MMP-9 activity respectively with progesterone compared to vehicle treated cells. Cocurrent treatment of cells with progesterone and calcitriol reduced the MMP-9 activity in HEC-1B (66%) and Ishikawa (68%) cells compared to vehicle treated cells (Figure 6A). These results showed further reduction of MMP-9 activity in HEC-1B (9%) and Ishikawa (6%) cells in response to combination treatment compared to progesterone alone. In both cell lines, activity of MMP-2 was significantly reduced (21–23%) in calcitriol treated cells. Progesterone alone exhibited 53% and 64% reduced MMP-2 activity in HEC-1B and Ishikawa cells respectively compared to vehicle treated cells. Treatment of cells with progesterone and calcitriol combination reduced MMP-2 activity by 63% in HEC-1B and 72% in Ishikawa cells compared to vehicle treated cells. These results revealed further reduction of MMP2 activity in HEC-1B (10%) and Ishikawa (8%) cells exposed to combination treatment compared to progesterone alone treated cells (Figure 6A).

**Figure 6:** Progesterone and calcitriol inhibit activity of MT1-MMP, MMP-9 and MMP-2 in cancer cells (**A**). HEC-1B and Ishikawa cells were treated with progesterone (PROG, 20 µmol/L), calcitriol (CAL, 100 nmol/L) or combination in the presence or absence of progesterone antagonist (RU 486) for 72 h were evaluated for activities of MT1-MMP, MMP-9 and MMP-2. Statistically significant changes in the treatment groups compared to their respective control groups are shown by asterisk (*P* < *0.05*). (**B**) Knockdown of ARF6 or NEDD9 in endometrial cancer cells resulted in decreased activities of MT1-MMP, MMP-9 and MMP-2. Statistically significant changes in the ARF6 and NEDD9 knockdown groups compared to their respective control groups are shown by asterisk (*P* < *0.05*).

The progesterone induced reduction of MT1-MMP, MMP-9 and MMP-2 activity was abrogated when cells were cultured with progesterone in the presence of progesterone receptor antagonist (RU 486). However, about 10–20% inhibition of MT1-MMP, MMP-9 and MMP-2 activity was seen when cells were cultured with calcitriol and progesterone-calcitriol combination in the presence of progesterone receptor antagonist (RU 486). These findings indicate that progesterone alone and progesterone-calcitriol combination are strong inhibitors and calcitriol is a moderate inhibitor of MT1-MMP, MMP-9 and MMP-2 activity in cancer cells.

### Depletion of ARF6 or NEDD9 alters activity of MT1-MMP

MT1-MMP plays an instrumental role in metastasis and both ARF6 and NEDD9 are promoters of tumorigenesis. We analyzed the activity of MT1-MMP, MMP-9 and MMP-2 in ARF6 or NEDD9 knockdown endometrial cancer cells and found significantly diminished activities of MT1-MMP, MMP-9 and MMP-2 compared to control siRNA transfected cells. These results suggest that ARF6 and NEDD9 are upstream of MT1-MMP and levels of ARF6 and NEDD9 modulate MT1-MMP activity and regulate cell invasiveness (Figure 6B).

### Progesterone and calcitriol inhibited expression of invadopodia related proteins in cancer cells

Cancer cell invasiveness and metastatic potential is dependent on the formation of invadopodia, which are actin-enriched membrane protrusions. To further investigate the effects of progesterone and calcitriol on the invasive potential of cancer cells, expression levels of invadopodia regulatory proteins (RAB-8, Rho A, cortactin, WIP, NWASP, and paxcillin) were assessed in endometrial cancer cells by Western blotting. Progesterone and the combination of calcitriol and progesterone markedly inhibited expression of all the proteins examined (Figure 7A). Inhibition was more pronounced with combination treatment than with progesterone alone. Additionally, correlation of these proteins with MT1-MMP expression was demonstrated by downregulation of RAB-8, cortactin, WIP, NWASP, paxcillin and Rho-A in MT1-MMP knockdown cells compared to scrambled siRNA cells (Figure 7B). These results suggest that progesterone-calcitriol inhibits invadopodia by downregulating MT1-MMP and reducing the expression of proteins involved in invadopodia formation (Figure 7B).

**Figure 7:** Knockdown of MT1-MMP reduced the expression of invadopodia related proteins (**A**) RAB 8, cortactin ,WIP, N-WASP and paxcillin levels were analyzed by Western blot analysis in progesterone, calcitriol or combination of two treated cell extracts or (**B**) cell lysates of MT1-MMP knockdown endometrial cancer cells. The values above the bands represent relative density of the bands normalized to β-actin.

## DISCUSSION

Cancer cell invasion and metastasis is a complex well-coordinated process, which involves rearrangement of cytoskeletal proteins resulting in extensive morphological changes. The membrane-anchored protein, MT1-MMP is an important regulator of cancer invasiveness and metastatic potential [31–34]. From the cell surface, MT1-MMP is internalized by clathrin-dependent or caveolar endocytic routes into endosomes, where it is either recycled back to the surface of the cell or moved to multivesicular bodies and lysosomes for degradation [22, 35]. The contribution of several proteins including NEDD9, ARF6, JIP3, JIP4 in the endocytosis and exocytosis of MT1-MMP is well established [26, 36, 37]. When cells are ready to migrate, MT1-MMP congregates to the front of cells in parallel with actin cytoskeleton and facilitates invadopodia formation. Exocytosis of MT1-MMP occurs at invadopodia, which extend into the extracellular matrix and mediate digestion and invasion through ECM [1]. Concentration of MT1-MMP in the invadopodia is accompanied with upregulation of multiple invadopodia proteins and increased cancer cell invasiveness [38].

ARF6, NEDD9 and MT1-MMP play an oncogenic role in tumor cell growth and are overexpressed in a variety of tumors [13, 14, 26, 39]. We compared the expression of ARF6, NEDD9 and MT1-MMP in normal endometrial tissues and in cancer patients. The three proteins were expressed at higher levels in the later stages of the disease. Our results concur with other studies which revealed positive correlation of ARF6, NEDD9 and MT1-MMP with advanced-stage disease and poor prognosis in solid tumors [14, 40–43]. We verified ARF6, NEDD9 and MT1-MMP expression patterns *in vitro* in an immortalized endometrial epithelial cell line (EM-E6/E7-TERT) and in endometrial cancer cell lines (HEC-1B, RL-95 and Ishikawa). These results corroborated the endometrial cancer tissue microarray results and are in accord with other studies exhibiting overexpression of these proteins in cancer cell lines [10, 42, 44, 45]. The results suggest that these proteins can be crucial biological markers of endometrial cancer invasion and metastasis. Knockdown of these proteins in HEC-1B and Ishikawa cells with specific siRNAs significantly suppressed invasive potential of cells, further substantiating their role in tumor aggressiveness. These findings are validated by other studies showing marked inhibition of gastric, breast, and cervical tumor migration and invasion by abrogation of ARF6, NEDD9 and MT1-MMP expression [14, 26, 39].

Our previous studies have shown that progesterone and calcitriol inhibit ovarian and endometrial cancer growth through caspase-3 activation, induction of G_0_–G_1_ cell-cycle arrest, downregulation of TGF-β, MMP-9 and MMP-2 signaling [27, 28, 29, 30]. In the present study, we found a moderate (10–20%) decrease of MT1-MMP activity in calcitriol treated cells compared to vehicle treated cells. However, the decrease was not observed when MT1-MMP expression was assessed using Western blotting. This discrepancy could be due to the sensitivity differences of the two assay systems. Previous studies have documented that progesterone, vitamin-D and its derivatives affect tumor invasion by decreasing the expression and activity of metalloproteinases; and by inducing their inhibitors [46–48]. A marked decrease of MT1-MMP, MMP-9 and MMP-2 activity was found in progesterone-calcitriol combination treated cells compared with progesterone or calcitriol alone treated cells. We have previously shown that progesterone enhances antitumorigenic actions of calcitriol in ovarian and endometrial cancer cells [29, 30] by inducing vitamin-D receptors on cancer cells and by inhibiting the expression of CYP24A1, an enzyme that catabolizes active vitamin-D. Together, our results presented in this study and previous studies suggest that synergistic effect of the two agents may have been related to the positive effect of progestins on vitamin-D activity.

However, the effect of progesterone and calcitriol on NEDD9 and ARF6 are not known. Here, we demonstrated a marked inhibition of ARF6, NEDD9 and MT1-MMP expression and activity of MT1-MMP with progesterone and calcitriol-progesterone combination treatment. Furthermore, the ARF6, NEDD9 and MT1-MMP suppression was abrogated in the presence of progesterone receptor antogonist, which delineates that major inhibitory effects are contributed via progesterone. These outcomes suggest an additional mechanism by which progesterone confers chemopreventive effects. Taken together, our data showed that ARF6, NEDD9 and MT1-MMP are involved in regulation of cell migration and invasion in endometrial cancer cells and silencing of these proteins by progesterone and calcitriol-progesterone treatment could be a promising approach for therapeutic intervention.

Our findings demonstrated inactivation of MT1-MMP in ARF6 and NEDD9 knockdown endometrial cancer cells compared to control siRNA transfected cells, implying that ARF6 and NEDD9 are upstream of MT1-MMP and modulators of MT1-MMP. Taken together, our results suggest a crucial role for ARF6 and NEDD9 as regulators of invasion in endometrial cancer through alteration of MT1-MMP activity, thus delineating an additional signaling pathway for targeting ARF6 and NEDD9 supported invasion. These findings concur with reports showing association of NEDD9 depletion with suppression of MT1-MMP mediated tumor cells invasion and metastasis in lung and breast cancers [26, 39].

Consistent with the expression of MT1-MMP on the cell surface and its critical role in cell invasion, the expression of MT1-MMP in endometrial cancer cells and its regulation with progesterone and calcitriol was investigated using immunofluorescence microscopy. Progesterone alone and in combination with calcitriol reduced the expression of MT1-MMP and translocated it to the cytoplasm, thus, abrogating the ability of cells to invade the ECM. Furthermore, progesterone and its combination with calcitriol, which also inhibits NEDD9 and ARF6, may disrupt MT1-MMP trafficking to the membrane. Taken together, our findings suggest that progesterone/calcitriol by depleting MT1-MMP from the cell surface while retaining it in the cytoplasm/endosome may serve as an effective inhibitor of tumor invasion and metastasis.

Invadopodia are actin-rich protrusions that are essential for invasion of cancer cells. There are three functional domains of invadopodia [49, 50]. The adhesive domain, consisting of several integrins, scaffold and signaling proteins, is involved in the adhesion of cells to the ECM and thus provides mechanical support to the invasive process. The proteolytic-domain participates in producing and transporting protease-containing vesicles to the invadopodia and degrades the ECM by metalloproteinases in concert with other proteins (RAB-8, RhoA). The invasive domain aids invadopodia in mechanical penetration into the ECM. It is composed of filamentous actin and a number of actin polymerization regulators (N-WASP, WIP, cortactin, Arp2/3 complex, cofilin, fascin). The small Rho-family GTPases are responsible for polymerization of actin by Arp2/3 complex via formation of N-WASP-WIP complex. Cortactin and facin reinforce and strengthen actin filaments and promote its penetration into the ECM. The cross-talk between the three domains orchestrates the invasion and migration of the cell into the matrix. The assembly of invadopodia is regulated by sequential interactions of several proteins. N-WASP, WIP, cortactin, RAB-8, Rho-A and paxcillin, proteins involved in distinct steps of invadopodia development, were detected in HEC-1B and Ishikawa cells. Treatment of cells with progesterone and calcitriol-progesterone combination effectively inhibited expression of invadopodia proteins and diminished invasive potential of cells.

In summary, our results suggest that in endometrial cancer ARF6 and NEDD9 proteins, which play a pivitol role in trafficking of MT1-MMP, are upregulated and as a consequence enhance the expression and presentation of MT1-MMP on cell surface (Figure 8). Increased concentration of MT1-MMP on the ventral cell surface initiates the formation of invadopodia by enhancing expression of the major constituents of invadopodia (matrix degrading enzymes, the actin-related proteins 2 and 3, WASP, N-WASP, WIP, cortactin, RAB-8, and, Rho A). The allows cells to direct extracellular matrix degradation and to facilitate cell migration across tissue microenvironment. Our findings suggest that progesterone-calcitriol treatment inhibits ARF6 and NEDD9 levels. In addition, progesterone-calcitriol translocates MT1-MMP from the cell surface into the cells. Hence, reduces the expression of invadopodia proteins and eventually suppresses cell invasiveness and metastasis. Thus, impediment of ARF6, NEDD9 and MT1-MMP interactions with progesterone-calcitriol may provide a therapeutic strategy for endometrial cancer treatment.

**Figure 8:** Model for progesterone-calcitriol mediated inhibition of MT1-MMP initiated invasive potential of cancer cells The model depicts that progesterone-calcitriol treatment inhibits expression of ARF6 and NEDD9, that are activated in cancer, and alters trafficking of activated MT1-MMP. Concentration of MT1-MMP on cell membrane initiates formation of invadopodia by stimulating invadopodia associated proteins. As a result of treatment, expression of ARF6, NEDD9 and MT1-MMP decreases and MT1-MMP relocates from cell surface to the cytoplasm. Consequently, expression of invadopodia associated proteins is reduced and formation is suppressed.

## MATERIALS AND METHODS

### Tissue microarrays (TMA) and immunohistochemistry (IHC)

The endometrial tissue microarrays (EMC1502) were purchased from US Biomax Inc.(Rockville, MD). The TMA contained normal [12], hyperplasia [3] and cancerous tissues of the endometrium in duplicates. After removal of paraffin from slides and quenching of endogenous peroxidase activity with 3% hydrogen peroxide, the slides were incubated with either ARF6 (1:200 dilution), NEDD9 (1:200 dilution), or MT1-MMP (1:100 dilution) antibodies for 18 h at 4C; followed by staining with secondary peroxidase-labeled antibodies and developed with DAB (Vector Laboratories Inc.). Positive and negative controls were included with each run. Staining was done in duplicate. Images were captured using a Nikon Eclipse E-800 microscope. The cores examined by two individuals for ARF6, NEDD9 and MT1-MMP staining intensity were categorized into four grades: 0, negative or trace amounts; 1, low; 2, medium; and 3, strong staining. The percentage of positively stained cells was grouped into four levels as follows: level 1 (< 25%); level 2 (25%–50%); level 3 (50%–75%); and level 4 (> 75%). For statistical determinations, final scores of 3 and 4 were defined as high expression and 1 and 2 scores as low expression. Staining intensity was quantified under high magnification (x20). The associations between ARF6, NEDD9 and MT1-MMP expression, tumor stage and grade were analyzed by Pearson’s chi-square (χ^2^) test. The percentage of cells expressing elevated levels of ARF6, NEDD9 and MT1-1MMP in endometrial tumors was high compared to normal endothelium. The differences were considered significant at a value of *p <0.05.*

### Cell lines and culture conditions

The human endometrial cancer cell lines HEC-1B and RL-95 were obtained from the American Type Culture Collection (ATCC) and Ishikawa cell line was obtained from Sigma. These cell lines were authenticated by DNA short-tandem repeat analysis by ATCC and Sigma. After purchasing, the cell lines were initially expanded and stored in multiple vials in liquid nitrogen. Cells were typically used for 3 months, at which time a fresh vial of cryopreserved cells was used. The HEC-1B and Ishikawa cells were grown in Eagle’s minimum essential medium (Invitrogen), and RL-95 were growth in Dulbecco’s Modified Eagle Medium (DMEM): Nutrient Mixture:F12 supplemented with 0.005 mg/mL Insulin (Invitrogen). Immortalized epithelial endometrial (EM-E6/E7-TERT) cells provided by Dr. Satoru Kyo (Kanazawa University, School of Medicine, Kanazawa, Japan) were grown in DMEM. All media were supplemented with 10% (v/v) FBS (Invitrogen), 100 U/mL penicillin, and 100 µg/mL streptomycin. The cells were cultured at 37^ο^C in a humidified atmosphere containing 5% CO_2_.

The cells were treated with progesterone (20 μmol/L PROG, 99.9% pure; Sigma), calcitriol (100 nmol/L; Sigma), or both for 72 hours and collected for protein extraction. The time of treatment and doses of progesterone and calcitriol were based on our previous studies showing inhibition of cell growth and apoptosis of cancer cells [27, 28, 29]. To test the specific effect of progesterone, cells were treated as stated above in the presence of progesterone receptor antagonist, mifepristone (0.1 mM, RU486, Sigma), to block the action of progesterone. For a set of experiments, HEC-1B and Ishikawa cells were seeded in 6-well plates and transfected the following day with siRNAs-targeting ARF6, NEDD9, MT1-MMP or scrambled siRNA (Santa Cruz Biotechnology and GE Dharmacon, Lafayette, CO) using the DharmaFECT transfection reagent (GE Dharmacon) for 48h and protein extracts were prepared for ARF6, NEDD9 and MT1-MMP analysis. The overall transfection efficiency for endometrial cells assessed by luciferase assay was 72% to 85%.

### Western blotting

Cells were lysed using a RIPA lysis buffer (Sigma). Equal amounts of protein from each sample were loaded onto the SDS-PAGE and then transferred to PVDF membranes (Thermo Fisher Scientific, Waltham, MA USA). After blocking with 5% nonfat milk in PBST for 1 h at room temperature, membranes were exposed to ARF6 (Santa Cruz Biotechnology, Inc Dallas, Texas), NEDD9 (Abcam, Cambridge, MA), MT1-MMP (Abcam.), RAB-8 (Cell Signaling Technology, Danvers, MA), Rho A, cortactin, WIP, paxcillin (Santa Cruz Biotechnology) NWASP (EMD MiIllipore, Billerica, MA) and β-actin (Sigma-Aldrich) antibodies. The enhanced chemiluminescence system was used to visualize the protein bands as recommended by the manufacturer (Thermo Fisher Scientific). Protein bands were quantified using densitometry software (Bio-Rad), and normalized using actin as a loading control. To calculate the relative intensity of each band, individual bands were divided by the corresponding loading control intensity.

### Invasion assay

ARF6, NEDD9, and MT1-MMP knocked down HEC-1B and Ishikawa cells and their scrambled siRNA transfected cells were used to assess the effects of knockdown of these proteins on the invasive property of endometrial cancer cells. The Biocoat Matrigel Invasion Chambers (BD Biosciences, San Jose, CA) were rehydrated at 37°C for 2 h. Control and knockdown cells were detached by trypsin and resuspended in serum-free medium. Medium containing 10% fetal bovine serum was applied to the lower chambers of BD BioCoat Matrigel Invasion Chambers as chemoattractant and then cells were seeded on the upper chambers at a density of 2.5 × 10^4^ cells/well in 100 ml of serum-free medium. The chambers were incubated for 16–18 h at 37°C. At 18 h after plating, noninvading cells were removed from the upper surface of the membrane by scrubbing. The cells on the lower surface of the membrane were fixed for 2 min in 100% methanol and stained with 1% toluidine blue in 1% sodium borate for 2 min. Cells that invaded through the insert were counted in five random fields per slide. All slides were coded to avoid biased counting. The assay was run in triplicates.

### MMP activity assays

MT1-MMP, MMP-9 and MMP-2 are the most crucial MMPs for the degradation of the ECM in cancers. The cell extracts of progesterone, calcitriol and progesterone-calcitriol combination treated HEC-1B and Ishikawa cells as well as extracts of ARF6 and NEDD9 knockdown cells were used to analyze the activities of MT1-MMP, MMP-9, and MMP-2. Changes in activity levels of three MMPs were determined using the SensoLyte 520 MMP-14, SensoLyte 520 MMP-9 and SensoLyte 520 MMP-2 assay kits from AnaSpec (San Jose, CA). Activities were assessed according to the manufacturer’s instructions. Briefly, specific respective substrates were added to samples and plates were incubated at 37°C for 30 to 60 min. Stop solution was added to each well and then fluorescence intensity was measured at excitation and emission wavelengths of 490 + 20 nm and 520 + 20 respectively. The fluorescence reading from the substrate control well was subtracted from the readings of the other wells. The fluorescence readings were expressed in relative fluorescence units (RFU). The RFU of control was considered as 100% and any change in samples was % change compared to control.

### Immunofluorescence microscopy

Endometrial cancer (HEC-1B and Ishikawa) cells seeded on coverslips were fixed in 4% paraformaldehyde for 20 minutes at room temperature and permeabilized with phosphatebuffered saline (PBS) containing 0.1% Triton X-100 (PBS-T) for 10 minutes, and subsequently blocked with PBS-T containing 5% normal goat serum for 1h. Cells were stained with MT1-MMP antibody (LifeSpan BioSciences Inc. Seattle, WA) for 1h in PBS-T containing 1% normal goat serum and a secondary antibody Alexa Fluor^®^ 488-labeled anti-mouse IgM antibody (Invitrogen Life Technologies). To detect F-actin, cells were stained with Phalloidin–Tetramethylrhodamine B isothiocyanate (Sigma-Aldrich) for 20 minutes and the cell nuclei were stained with 1µg/mL DAPI for 10 minutes. Fluorescent images of cells were captured using a LSM 710 laser scanning confocal microscope (Carl Zeiss Microscopy, LLC Thornwood NY). Quantitative analysis of confocal z-stacks was executed using Image J software. The cell outlines from the projected z-stacks were drawn in random fields and the sum of the pixel values within the outlines in the MT1-1MMP channel was ascertained and the background was subtracted which represents MT1-MMP fluorescence within the cell. In each group 30 cells were assessed for fluorescence intensity. Statistical analysis was performed using a two-sided Fisher’s test.

### Statistical analysis

The data were representative of three independent experiments as the mean ± SEM. Statistical significance was assessed using one-way analysis of variance and Student’s unpaired *t* test. *P*-value < 0.05 was considered significant.

## DISCLAIMER

The opinions or assertions contained herein are the private views of the authors and are not to be construed as official or as reflecting the views of the Uniformed Services University of the Health Sciences, the Department of the Air Force, the Department of the Army, the Department of the Navy, or the Department of Defense.
